The article "Effect of different anesthetic methods on cellular immune functioning and the prognosis of patients with ovarian cancer undergoing oophorectomy" was retracted in 2022. Reasons: false authorship; concerns about the authorship.

# Effect of different anesthetic methods on cellular immune functioning and the prognosis of patients with ovarian cancer undergoing oophorectomy

**DOI:** 10.1042/BSR20170915

**Published:** 2017-10-24

**Authors:** Xin-Rui Han, Xin Wen, Yan-Yi Li, Shao-Hua Fan, Zi-Feng Zhang, Hong Li, Xing-Feng Sun, Gui-Qi Geng, Shen Sun, Shao-Qiang Huang, Dong-Mei Wu, Jun Lu, Yuan-Lin Zheng

**Affiliations:** 1 Key Laboratory for Biotechnology on Medicinal Plants of Jiangsu Province, School of Life Science, Jiangsu Normal University, Xuzhou 221116, P.R. China; 2 Department of Gynecology and Obstetrics, Shanghai Pudong Hospital, Fudan University Pudong Medical Center, Shanghai 201399, P.R. China; 3 Department of Anesthesiology, Obstetrics & Gynecology Hospital of Fudan University, Shanghai 200090, P.R. China

**Keywords:** Combined general/epidural anesthesia, cellular immune function and prognosis, general anesthesia, ovarian cance

## Abstract

The present study aimed to explore the effects of different anesthetic methods on cellular immune function and prognosis of patients with ovarian cancer (OC) undergoing oophorectomy. A total of 167 patients who received general anesthesia (GA) treatment (GA group) and 154 patients who received combined general/epidural anesthesia (GEA) treatment (GEA group) were collected retrospectively. Each group selected 124 patients that met the inclusion and exclusion criteria for further study. ELISA and radioimmunoassay were employed to detect levels of IL-2, TNF-α, and CA-125. The rates of tumor-red cell rosette (RTRR), red cell immune complex rosette (RRICR), and red cell C3b receptor rosette (RRCR) were also measured. Systolic blood pressure (SBP), diastolic blood pressure (DBP), and heart rate (HR) were determined by hemodynamics. The levels of tumor necrosis factor-α (TNF-α) and interleukin (IL)-2 decreased at 1 h intraoperation (T2), but increased 24-h post surgery (T3). The levels of TNF-α and IL-2 were recovered faster in the GEA group than in the GA group. The GA group exhibited greater levels of CA-125 expression than in the GEA group. The levels of RTRR, RRICR, and RRCR; ratios of CD3^+^, CD4^+^, CD4^+^/CD8^+^, CD16^+^, and CD56^+^ at 30 min after anesthesia (T1), T2, T3 and 48 h after the operation (T4) and levels of SBP, DBP, and HR at T1, T2, and T3 displayed increased levels in the GEA group than in the GA group. At 72-h post surgery (T5), the 5-year survival rate significantly increased in the GEA group compared with the GA group. GEA to be more suitable than GA for surgery on OC patients.

## Introduction

Ovarian cancer (OC), a gynecological cancer widely considered a primary gynecological malignancy with a 5-year survival rate of 25–35% [1,2]. Worldwide, OC currently ranks as the seventh leading cancer diagnosis as well as the eighth foremost cause of cancer mortality [3]. OC is characterized by several nonspecific symptoms such as dyspepsia, abdominal discomfort including fullness, and bloating [4]. The symptoms of OC at the early stages are generally absent, which makes diagnoses in its early stages exceedingly difficult [5]. In regards to treatments, surgery and chemotherapy are often selected for OC patients; however, it is estimated that 70–75% of all women suffering from OC will experience a recurrence [6]. Laparoscopy is considered to be a minimally invasive and cost-effective surgical procedure capable of reducing postoperative pain, urinary tract infection, and managing ovarian neoplasms [7]. However, the respective method of anesthesia selected is associated with the risk of surgery [8]. Therefore, it is of great importance to evaluate the effects of different anesthetic methods on OC patients.

General anesthesia (GA) is a controlled unconsciousness state where gaseous or intravenous drugs are used to depress a patient’s central neurological system in order to eliminate their protective reflexes [9,10]. GA is known to cause surgical stress and may directly activate the sympathetic nervous system, the hypothalamic–pituitary–adrenal axis as well as affect the immune system [11]. Epidural anesthesia is able to ease severe pain by reducing respiratory and cardiovascular complications, in addition to being supportive of early mobilization post surgery [12]. Combined general/epidural anesthesia (GEA) methods are frequently used anesthetic techniques in abdominal or thoracic surgical contexts. GEA can influence cerebral hemodynamics, intracranial pressure, and adverse cerebrovascular responses in patients undergoing laparoscopic procedures [7]. All methods of anesthesia elicit some effects on the individual’s cellular immunity through immune competent cells in a directly suppressive manner. This is especially the case in cancer patients with severe immunosuppression by anesthesia and dysfunction of natural killer (NK) cells. Metastasis accounts for the principal cause of death in regards to ovarian cancer patients [13]. Immunosuppression may promote the metastases and growth of residual malignant cells and worsen prognosis [11]. Thus, the present study aimed to investigate the effects of both GA and GEA on cellular immune functioning, as well as the prognosis of OC patients.

## Method and materials

### Ethics statement

The study was conducted under the approval of the Clinical Trials Ethics Committee of Shanghai Pudong Hospital, Fudan University Pudong Medical Center. All participating patients signed informed consent documentation.

### Study subjects and grouping

Case notes of 167 patients who received GA treatment and 154 patients who received GEA treatment between July 2012 and July 2015 were collected retrospectively. Patients were aged between 18 and 77 years old, who had been treated in the gynecology department of Obstetrics & Gynecology Hospital of Fudan University. A total of 167 patients who received GA treatment (GA group) and 154 patients who received GEA treatment (GEA group) were collected retrospectively. Each group selected 124 patients that met the inclusion and exclusion criteria for further study. The double-blind method was adopted for the experiments, and test subjects, test implementers, and outcome measurers were not privy to information regarding where the subjects were assigned. All selected patients had been diagnosed with malignant epithelial tumors based on the histological classification of ovarian tumors established by the World Health Organization (WHO) [14]. None of the patients had previously undergone any previous operative treatments or chemotherapy. Staging was carried out based on the International Federation of Gynecology and Obstetrics (IFGO) [15] staging criteria. The inclusion criteria were as follows: (1) all patients had been confirmed pathologically as epithelial EC patients and underwent laparoscopic surgical treatment at the gynecology department of Shanghai Pudong Hospital, Fudan University Pudong Medical Center; (2) patients who had complete clinical and follow-up data; (3) patients who were verified to have a malignant epithelial tumor. The exclusion criteria were as follows: (1) patients were diagnosed with other malignant tumors; (2) patients were at the time of examination advanced OC cases or had previously undergone operative treatment or chemotherapy; (3) patients who did not have sex cord-stromal tumors, germ cell tumors, or any other mixed type of tumor; (4) patients did not have borderline tumor.

### Anesthesia regimen, surgical treatment, and postoperative analgesia method

All patients were administered intramuscular injections of 0.5 mg of atropine and 0.1 g of phenobarbital sodium and intravenously injected with lactated Ringer’s solution 30 min before their respective operations. In the GA group, an intravenous drip containing 0.5 mg/kg of midazolam (batch number: 20160411, Jiangsu Nhwa Pharmaceutical Corporation Ltd., Jiangsu, China), 0.5 μg/kg of sufentanyl (batch number: H1161002, Yichang Humanwell Pharmaceutical Co., Ltd., Hubei, China), 0.15 mg/kg of cisatracurium (batch number: 16101418, Jiangsu Hengrui Medicine co., Ltd, Jiangsu, China), and 1.5 mg/kg of propofol (batch number: MG042, AstraZeneca, UK Limited, London, U.K.) was given to each patient. Following the introduction of anesthesia, a trachea cannula was inserted. Propofol [6–10 mg/(kg·h)] was continuously administered drip-wise while sulfentanyl and cisatracurium were intermittently injected throughout the operation. Patients in the GEA group were injected with 3 ml of 2% lidocaine and anesthesia introduction was performed following the determination of the block level. Patients then had a trachea cannula implanted. A solution consisted of 3–6 mg/(kg·h) of propofol was continuously injected and 0.75% ropivacaine (6–8 ml/h) was injected into the epidural space. OC patients at an early OC stage underwent laparoscopic OC tumor resection. During the operation, blood oxygen saturation, electrocardiogram readings, and intra-airway pressure were all closely monitored. The trocar was rotated to puncture the abdomen 10 mm over the navel (confirmed by the accessed lens). Artificial pneumoperitoneum was established by filling CO_2_, and cancer cells were examined using conventional cytology. The omentum majus was resected using an ultrasound knife and the pelvic cavity and the abdominal para-aortic lymph nodes were cleaned. The uterus, fallopian tubes, and ovaries were also removed using an ultrasound knife and then appendectomy and wound hemostasis were conducted respectively. Sterile water was used to clean the pelvic cavity and puncture sites where drainage tubes were placed. The potency ratio between sufentanil and fentanyl was 1:10. The laparoscopic cytoreductive surgery could potentially be adapted according to the disease severity of OC patients. In specific terms, the radical pelvic resection, intestinal resection, diaphragm, or other peritoneal surface dissection; splenectomy, partial hepatectomy, cholecystectomy, partial gastrectomy, or cystectomy; uerterovesicostomy, distal pancreatectomy, or appendectomy could be conducted based on clinical features and conditions. Patients in the GA and GEA groups were administered 2 mg of 0.25% bupivacaine and morphine (6 ml in total) after surgery, and an extradural injection was administered 0.5 h prior to abdominal closure. Subsequently, 100 ml of 0.125% bupivacaine and morphine [0.06 mg/(kg/d)] was administered at a constant rate of 2 ml/h for 2 days via extradural injection.

### Postoperative treatment

Following the operative procedure, patients received routine prophylactic anti-infection and fluid replacement for symptomatic treatment purposes. Patients in both groups were given small liquid diets 1 day after undergoing their respective procedures. According to the routine pathology examination and surgical/pathologic-stage results, patients at grade 1 (G1) of international federation of gynecology and obstetrics (FIGO) stage IA and IB were those that displayed good prognosis did not receive chemotherapy treatment. Patients at G2 and G3 of FIGO stage IA and IB patients, or patients with clear-cell carcinoma or patients at stage IC were given 4–6 courses of chemotherapy with paclitaxel and platinum following their surgical procedure. Chemotherapy was not conducted until patient’s normal routine blood test results had been confirmed, stable vital signs and normal gastrointestinal and urinary system functioning were observed.

### Observation of intraoperative and postoperative indexes

The operation time was defined as the time span between the very first skin incision until the end of surgery. Intraoperative blood loss was defined as the volume of blood lost measured by the anesthetist after surgery. Hospitalization time was time span from the day after surgery to the day the patient was released from the hospital after complete recovery. Postoperative fart time was the time after which normal intestinal peristalsis was recovered (passage of gas by anus as the symbol). Postoperative infection was defined as oozing from the surgical wound or purulent secretion. Indolence, nonhealing, and postoperative hypotension were defined as systolic pressure (high pressure) lower than 100 mmHg or diastolic pressure (low pressure) lower than 60 mmHg. Rehospitalization was understood to be a scenario in which patients were readministered to the hospital after surgery as well as patients readmitted to the hospital after the follow-up period had ended.

### Sample collection and enzyme-linked immunosorbent assay (ELISA)

A total of 5 ml of venous blood was collected from every patient in the GA and GEA groups at six different time points: before anesthesia (T0), 30 mins after anesthesia (T1), 1 h intraoperation (T3), 24 h after the operation (T3), 48 h after the operation (T4), and 72 h after the operation (T5). The respective samples were piped into heparinized anticoagulation tubes. A total of 2 ml of whole blood was also collected at each time point and centrifuged for 5 mins at 500–1000 r/min. Plasma was obtained and ELISA (Wuhan Boster Biological Technology Ltd., Hubei, China) was employed to detect the levels of interleukin (IL)-2 and tumor necrosis factor-α (TNF-α) in accordance with the kit instructions. When both the reaction and coloration had been terminated, the optical density (OD) value was obtained at a wavelength of 150 nm using an enzyme-labeled meter. Standard concentration represented the horizontal ordinate, while the OD value of 450 nm was the vertical coordinate. SPSS16.0 software (IBM-SPSS Inc., Chicago, IL, U.S.A.) was used to draw the standard curves.

### Radioimmunoassay

Serums from all OC patients from both groups were obtained at T0 and T1. In accordance with the instructions of CA-125 kit (Art. No. ML-(E)-a3525, Shanghai Enzyme-linked Biotechnology Co., Ltd., Shanghai, China), a radioimmunoassay was used to detect the expression of CA-125 before and after anesthesia.

### Red blood cell immune complex (RBC-IC) rosette test

Three milliliters of anticoagulated whole blood was obtained at each time point and centrifuged for 10 min at 3000 r/min to separate the upper layer plasma from red blood cells. The separated plasma was stored at 4°C for further use. The red blood cells were washed three times using normal saline solution at a ratio of 1:3. The supernatant was subsequently discarded after centrifugation. Red blood cell suspension was obtained (ratio of red blood cells to normal saline at 1:1) and stored at 4°C for further use. Human OC cells, purchased from American Tissue Culture Collection (ATCC, Manassas, VA, U.S.A.), were washed twice with normal saline and then suspended with phosphate-buffered saline (PBS, Wuhan Boster Biological Technology Co., Ltd., Hubei, China) at a cell density of 1 × 10^6^/ml. A total of 150 μl of cell suspension was mixed with an equal volume of plasma and placed in a 37°C water bath for 1 h. The mixture was then centrifuged, washed twice, and the supernatant was discarded. Sensitive cancer cells (induced by a serum) were obtained, mixed with 50 μl of red blood cell suspension, and placed in a water bath at 37°C for 45 min. Glutaraldehyde (0.05%) was added to fix and smear the solution. Finally, Wright’s staining method was performed (Wuhan Boster Biological Technology Ltd., Wuhan, Hubei, China). Tumor-red cell immune rosette was defined as a tumor cell combined with three or more red blood cells. A total of 100 tumor cells were observed and counted under an oil immersion lens, and the rate of tumor-red cell rosette (RTRR) was subsequently calculated. Yeast suspension was obtained by mixing yeast polysaccharides under 37°C conditions. Plasma (150 μl) was added to 150 μl of saccharomycetes suspension and water bathed at 37°C for 30 min. Similarly, the rate of red cell immune complex rosette (RRICR) and rate of red cell C3b receptor rosette (RRCR) too was calculated.

### Flow cytometry

A total of 0.1 ml of anticoagulated whole blood was obtained the previously discussed time point and centrifuged. The lower layer red blood cells (50 μl) were washed three times with PBS followed by centrifugation and removal of the supernatant. Red blood cell suspension was then made by mixing red blood cells with PBS and divided into five separate test tubes (100 μl/per tube). Subsequently, 0.01 ml of monoclonal antibody marked by cluster of differentiation 3 (CD3) peridinin chlorophyll protein (PerCP), CD4 fluorescein isothiocyanate (FITC), CD8 phycoerythrin (PE) and monoclonal antibody (Beckman Coulter, Inc., Fullerton, CA, U.S.A.), and labeled by CD16 FITC and CD56 PE were added, thoroughly mixed followed by incubation for 30 min at room temperature under dark conditions. The mixture was then washed with 1 ml of PBS, centrifuged, and then the supernatant was discarded. Another 500 μl of PBS was added, thoroughly mixed and then the flow cytometer (Beckman Coulter, Inc., Fullerton, CA, U.S.A.) was used for detection purposes.

### Detection of systolic blood pressure (SBP), diastolic blood pressure (DBP), and heart rate (HR)

The SBP, DBP, and HR of OC patients were observed at the following time points: before anesthesia (T0), 30 min after anesthesia (T1), 1-h intraoperation (T2), 24 h after operation (T3), 48 h after operation (T4), and 72 h after operation (T5). The SBP, DBP, and HR values of patients in the GA and GEA groups were compared at each time.

### Visual analog scale (VAS) score

The visual analog scale (VAS) score was calculated for all patients before operation and 72 h after their respective procedures. First, the use of the VAS score was explained to all patients in detail to ensure each patient was well aware of the objective in order to ensure accuracy. Patients were then self-evaluated based on their degree of pain. A 10 cm long and 2-finger wide hardboard was selected for the experiment. On one side, there was no scale and just one black line in the middle of the board. On the other side, there were different scales ranging from 0 to 10. On the hardboard, 0 represented no pain, while 0–3 represented slight but tolerable pain, 4–6 represented pain that was tolerable but had an effect on sleep, and 7–10 represented intolerable or severe pain that affected both appetite and sleep. All scores from the results were recorded in detail.

### Follow-up

Patients in both groups were followed-up every month following their respective operative procedures as well as chemotherapy. The follow-up period lasted 5 years. In the event that a patient passed away or was not able to be contacted, the follow-up process was abandoned. Detailed information regarding the follow-up and clinical data of OC patients in both groups were recorded. Survival curves were drawn to analyze the survival rates of OC patients in both the GA and GEA groups.

### Statistical analysis

All data were analyzed using the SPSS18.0 software (IBM Corp. Armonk, NY, U.S.A.). Measurement data were represented as mean ± standard deviation (SD). Normal distributions were compared using unpaired and paired *t*-tests. Comparison among multiple groups was conducted via one-way analysis of variance (ANOVA), while comparisons between two groups were performed using a fisher’s least significant difference (LSD) test. Measurement data without normal distribution were compared using a rank-sum test. Furthermore, the comparison of cytokine concentrations was detected using the variance of repeated measured data. Enumeration data were represented as a percentage or ratio and the chi-square test was used for comparisons. *P*<0.05 was indicative of statistical significance.

## Results

### Baseline characteristics of the GA and GEA groups

Study subjects in the GA (*n*=124) and GEA (*n*=124) groups were all anesthetized at the gynecology department of Shanghai Pudong Hospital, Fudan University Pudong Medical Center. All patients underwent laparoscopic tumor resection procedures. There were no significant differences detected regarding age, menopause, tumor diameter, history of abdominal surgery, complications, pathological type, clinical stage as well as tumor grade between the GA and GEA groups (all *P*>0.05, Table 1). All data collected from both groups were comparable.

**Table 1:** Comparisons of baseline characteristics between the GA and GEA groups

Baseline characteristic	GA group (*n*=124)	GEA group (*n*=124)	*P*
Age (years)	42.28 ± 8.44	43.03 ± 8.93	0.497
Menopause [*n* (%)]	41 (33.1)	45 (36.3)	0.594
Tumor diameter (cm)	8.73 ± 0.72	8.97 ± 0.58	0.117
History of abdominal surgery [*n* (%)]	47 (37.9)	45 (36.3)	0.793
Complication [*n* (%)]	14 (11.3)	18 (14.5)	0.449
Pathological type			0.915
Serous papillary carcinoma [*n* (%)]	33 (26.6)	37 (29.8)	
Mucoid adenocarcinoma [*n* (%)]	19 (15.3)	16 (12.9)	
Endometrioid adenocarcinoma [*n* (%)]	27 (21.8)	24 (19.4)	
Clear-cell carcinoma [*n* (%)]	25 (20.2)	29 (23.4)	
Transitional cell carcinoma [*n* (%)]	9 (7.3)	10 (8.1)	
Other types [*n* (%)]	11 (8.9)	8 (6.5)	
Clinical stage			0.549
I [*n* (%)]	16 (12.9)	18 (14.5)	
II [*n* (%)]	22 (17.7)	26 (21.0)	
III [*n* (%)]	33 (26.6)	40 (32.3)	
IV [*n* (%)]	53(42.7)	40 (32.3)	
Tumor grade			0.811
G1grade (well-differentiated tumor)	9 (7.2)	8 (6.5)	
G2 grade (middle-differentiated tumor)	44 (35.5)	40 (32.3)	
G3 grade (poorly differentiated tumor)	71 (57.3)	76 (61.3)	

Notes: Complication, in the general anesthesia group, hypertension (*n*=9), hypertension complicated with arrhythmia (*n*=5); in the combined general/epidural anesthesia group, hypertension (*n*=12), hypertension complicated with arrhythmia (*n*=5), diabetes (*n*=1); Abbreviations: GA, general anesthesia; GEA, combined general/epidural anesthesia.

### Comparison of intraoperative and postoperative indexes in the GA and GEA groups

There were no significant differences in the operative time, intraoperative blood loss, and hospitalization time of the GA and GEA groups (*P*>0.05). However, postoperative fart time and rates of postoperative infection, postoperative hypotension, and rehospitalization showed significant differences (*P*<0.05) (Table 2).

**Table 2:** Comparisons of intraoperative and postoperative parameters between the GA and GEA groups

Parameter	GA group (*n*=124)	GEA group (*n*=124)	*P*
Operative time (min)	267.4 ± 45.2	271.8 ± 51.6	0.476
Intraoperative blood loss (ml)	156.34 ± 45.3	167.32 ± 51.8	0.077
Hospitalization time (d)	13.6 ± 3.5	13.1 ± 4.2	0.31
Postoperative fart time (d)	3.4 ± 1.3	1.5 ± 0.8	<0.001
Postoperative infection [*n* (%)]	23 (18.5)	9 (7.3)	0.008
Postoperative hypotension [*n* (%)]	21 (16.9)	7 (5.6)	0.005
Rehospitalization [*n* (%)]	16 (12.9)	6 (4.8)	0.026

Abbreviations: GA, general anesthesia; GEA, combined general/epidural anesthesia.

### Levels of IL-2 and TNF-α at various time points in the GA and GEA groups

Both the levels of IL-2 and TNF-α exhibited slight decreases at T1, which was significantly further reduced at T2 compared with T0 (*P*<0.05). After T3, their expressions displayed gradually up-regulated levels. Compared with T0, the levels of IL-2 and TNF-α in the GA group were reduced at T3 and T4 (*P*<0.05) with no significant difference detected at T5 (*P*>0.05). While in the GEA group, the levels of IL-2 and TNF-α exhibited down-regulated levels at T3 (*P*<0.05), and no differences were detected at T4 and T5 (*P*>0.05). The results illustrated quicker recovery of IL-2 and TNF-α levels in the GEA group than in the GA group. Compared with patients in the GEA group, patients in the GA group displayed no obvious differences regarding the serum levels of IL-2 and TNF-α at T0 and T5 (both *P*>0.05); however higher levels were observed at T2, with lower levels detected at T3 and T4 (all *P*<0.05, Table 3).

**Table 3:** Comparisons of the levels of IL-2 and TNF-α in the GA and GEA groups

Groups	Immune factors	T0	T1	T2	T3	T4	T5
The GA group	IL-2 (pg/ml)	5.09 ± 0.42	5.03 ± 0.38	4.13 ± 0.34*^†^	4.24 ± 0.56*^†^	4.32 ± 0.63*^†^	5.05 ± 0.69
	TNF-α (pg/ml)	30.17 ± 3.16	30.13 ± 3.12	28.18 ± 2.58*^†^	28.34 ± 2.67*^†^	28.78 ± 2.74*^†^	30.05 ± 3.12
The GEA group	IL-2 (pg/ml)	5.13 ± 0.45	5.06 ± 0.43	3.94 ± 0.39^†^	4.47 ± 0.71^†^	5.17 ± 0.75	5.19 ± 0.77
	TNF-α (pg/ml)	30.58 ± 3.21	30.56 ± 3.19	27.16 ± 2.83^†^	29.45 ± 3.01^†^	29.43 ± 3.32	30.62 ± 3.22

Notes: *, compared with the GEA group, *P*<0.05; †, compared with T0, *P*<0.05; Abbreviations: GA, general anesthesia; GEA, combined general/epidural anesthesia; IL-2, interleukin-2; TNF-α, tumor necrosis factor-α.

### Comparisons of CA-125 expression at different time points in the GA and GEA groups

There was no difference detected in relation to expressions of C-125 in the GA and GEA groups at T0 (*P*>0.05). Furthermore, the GEA group exhibited higher CA-125 expression than the GA group at T5 (Table 4).

**Table 4:** CA-125 expression in serum before and after anesthesia in the GA and GEA groups

	T0	T5
GA group	245.93 ± 45.26 U/ml	158.94 ± 36.18 U/ml*
GEA group	252.67 ± 53.24 U/ml	133.57 ± 27.24 U/ml

Notes: *, compared with the GEA group, *P*<0.05; Abbreviations: GA, general anesthesia; GEA, combined general/epidural anesthesia.

### RTRR, RRICR, and RRCR at different time points in the GA and GEA groups

RTRR, RRICR, and RRCR were significantly lower at T1, T2, and T3 than at T0 in the GA and GEA groups (all *P*<0.05). At T4, RTRR, RRICR, and RRCR in both groups began to increase. Statistically significant differences were detected at T1, T2, T3, and T4 compared with T0. There was no obvious difference in relation to RTRR, RRICR, and RRCR at T0 and T5 between the two groups (all *P*>0.05). At T1, T2, T3, and T4 and RTRR, RRICR, and RRCR in the GA group were significantly lower than in the GEA group (all *P*<0.05) (Table 5).

**Table 5:** Comparisons of RTRR, RRICR, and RRCR between the GA and GEA groups

	Group	T0	T1	T2	T3	T4	T5
RTRR	GA group	24.37 ± 1.91	19.52 ± 1.36*^†^	19.22 ± 1.31*^†^	18.75 ± 1.27*^†^	19.81 ± 1.37*^†^	24.26 ± 1.81
	GEA group	24.71 ± 1.98	22.13 ± 1.62^†^	21.64 ± 1.55^†^	21.15 ± 1.42^†^	22.07 ± 1.73^†^	24.53 ± 1.85
RRICR	GA group	46.08 ± 3.72	30.26 ± 3.05*^†^	29.32 ± 3.03*^†^	29.01 ± 2.95*^†^	30.34 ± 3.19*^†^	45.11 ± 3.67
	GEA group	46.25 ± 3.77	33.84 ± 3.61^†^	33.47 ± 3.55^†^	32.84 ± 3.47^†^	33.96 ± 3.59^†^	45.99 ± 3.69
RRCR	GA group	47.62 ± 3.93	39.65 ± 3.67*^†^	38.94 ± 3.58*^†^	37.86 ± 3.53*^†^	39.71 ± 3.71*^†^	46.75 ± 3.91
	GEA group	47.83 ± 3.96	42.17 ± 3.85^†^	41.88 ± 3.81^†^	41.59 ± 3.77^†^	42.19 ± 3.89^†^	46.92 ± 3.93

Notes: *, compared with the GEA group, *P*<0.05; †, compared with T0, *P*<0.05; Abbreviations: GA, general anesthesia; GEA, combined general/epidural anesthesia; RRCR, rate of red cell C3b receptor rosette; RRICR, rate of red cell immune complex rosette; RTRR, rate of tumor-red cell rosette.

### The ratio of CD3^+^, CD4^+^, CD4^+^/CD8^+^, CD8^+^, CD16^+^, and CD56^+^ at different time points in the GA and GEA groups

The ratios of CD3^+^, CD4^+^, CD4^+^/CD8^+^, CD16^+^, and CD56^+^ at T1, T2, T3, and T4 were all lower than the observed ratios at T0 in both the GA and GEA groups (all *P*<0.05). The above parameters began to increase at T4 in both groups. There was no significant difference in the ratios of CD3^+^, CD4^+^, CD4^+^/CD8^+^, CD16^+^, and CD56^+^ at T0 and T5 between the two groups (all *P*>0.05). At T1, T2, T3, and T4, the ratios of CD3^+^, CD4^+^, CD4^+^/CD8^+^, CD16^+^, and CD56^+^ in the GA group were significantly lower than those in the GEA group (*P*<0.05, Table 6). There was no apparent difference regarding the ratio of CD8^+^ at any time point in both groups (all *P*>0.05).

**Table 6:** Comparisons of ratios of CD3^+^, CD4^+^, CD4^+^/CD8^+^, CD8^+^, and NK cells between the general anesthesia (GA) and combined general/epidural anesthesia (GEA) groups

Time	Group	CD3^+^ (%)	CD4^+^ (%)	CD8^+^ (%)	CD4^+^/CD8^+^ (%)	NK (%)
T0	GA group	64.37 ± 6.71	35.02 ± 3.11	26.84 ± 2.49	1.30 ± 0.22	8.03 ± 0.78
	GEA group	64.55 ± 6.73	35.11 ± 3.14	27.02 ± 2.58	1.30 ± 0.25	8.18 ± 0.82
T1	GA group	55.89 ± 6.18*^†^	27.60 ± 2.66*^†^	26.69 ± 2.41	1.03 ± 0.19*^†^	5.78 ± 0.59*^†^
	GEA group	60.23 ± 6.25^†^	31.72 ± 2.94^†^	26.91 ± 2.53	1.15 ± 0.22^†^	6.95 ± 0.68^†^
T2	GA group	56.61 ± 6.14*^†^	27.48 ± 2.61*^†^	26.57 ± 2.36	1.03 ± 0.14*^†^	5.74 ± 0.55*^†^
	GEA group	60.02 ± 6.21^†^	31.51 ± 2.90^†^	26.85 ± 2.49	1.17 ± 0.17^†^	6.91 ± 0.61^†^
T3	GA group	53.03 ± 6.02*^†^	27.92 ± 2.57*^†^	26.51 ± 2.32	1.13 ± 0.11*^†^	5.56 ± 0.47*^†^
	GEA group	59.88 ± 6.19^†^	31.32 ± 2.84^†^	26.79 ± 2.45	1.17 ± 0.15^†^	6.89 ± 0.59^†^
T4	GA group	55.11 ± 6.18*^†^	28.11 ± 2.73*^†^	26.82 ± 2.44	1.05 ± 0.14*^†^	5.69 ± 042*^†^
	GEA group	59.79 ± 6.34^†^	31.37 ± 2.91^†^	26.87 ± 3.01	1.17 ± 0.19	6.90 ± 0.56^†^
T5	GA group	63.34 ± 6.51	34.02 ± 3.04	26.95 ± 2.51	1.26 ± 0.18	7.93 ± 0.72
	GEA group	63.50 ± 6.62	34.29 ± 3.08	27.01 ± 2.55	1.27 ± 0.21	8.02 ± 0.80

Notes: *, compared with the GEA group, *P*<0.05; †, compared with T0, *P*<0.05; Abbreviations: CD, cluster of differentiation; GA, general anesthesia; GEA, combined general/epidural anesthesia; NK, natural killer.

### The levels of SBP, DBP, and HR at different time points in the GA and GEA groups

The levels of SBP, DBP, and HR at T1, T2, and T3 were all significantly lower than those at T0 in both the GA and GEA groups (all *P*<0.05). The levels of SBP, DBP, and HR began to increase at T4 in both groups. There was no significant difference detected in the levels of SBP, DBP, and HR at T0, T4, and T5 between two groups (all *P*<0.05). However, the GA group had lower levels of SBP, DBP, and HR than the GEA group at T1, T2, and T3 (all *P*<0.05, Table 7).

**Table 7:** Comparisons of SBP, DBP, and HR between the general anesthesia (GA) and combined general/epidural anesthesia (GEA) groups

Group	Index	T0	T1	T2	T3	T4	T5
GA group	SBP	116.2 ± 9.5	108.6 ± 8.9*^†^	108.4 ± 8.6*^†^	107.8 ± 8.5*^†^	113.5 ± 9.1	113.9 ± 9.4
	DBP	66.8 ± 7.3	60.4 ± 6.7*^†^	59.8 ± 6.5*^†^	59.1 ± 6.2*^†^	64.5 ± 6.9	64.9 ± 7.1
	HR	75.7 ± 7.8	70.2 ± 7.4*^†^	69.8 ± 7.1*^†^	69.5 ± 6.8*^†^	73.9 ± 7.2	74.3 ± 7.5
GEA group	SBP	118.8 ± 9.7	113.9 ± 9.5^†^	113.3 ± 9.3^†^	112.7 ± 9.1^†^	115.5 ± 9.2	116.1 ± 9.7
	DBP	68.3 ± 7.5	63.8 ± 7.1^†^	63.5 ± 6.9^†^	63.2 ± 6.7^†^	65.8 ± 7.2	66.4 ± 7.4
	HR	77.9 ± 7.8	74.0 ± 7.6^†^	73.8 ± 7.5^†^	73.4 ± 7.3^†^	75.2 ± 7.6	76.7 ± 7.7

Notes: *, compared with the GEA group, all *P*<0.05; †, compared with T0, *P*<0.05; Abbreviations: DBP, diastolic blood pressure; GA, general anesthesia; GEA, combined general/epidural anesthesia; HR, heart rate; SBP, systolic blood pressure.

### VAS score before operation and 72 h after operation in the GA and GEA groups

The VAS scores prior to the operative procedure as well as 72-h post surgery were significantly different in the GA and GEA groups (all *P*<0.05). However, there was no significant difference detected regarding the VAS score between the GA and GEA groups (all *P*>0.05). The VAS score in the GEA group 72 h after the operative procedures was lower than that in the GA group (*P*<0.05, Table 8).

**Table 8:** Comparison of VAS score before and 72 h after operation between GA and GEA groups

Group	Before operation	72 h after operation
GA group	7.76 ± 0.48	5.64 ± 0.35*^†^
GEA group	7.72 ± 0.46	3.31 ± 0.32^†^

Notes: *, compared with the combined GEA group, all *P*<0.05; ^†^, compared with preoperation, *P*<0.05; Abbreviations: GA, general anesthesia; GEA, combined general/epidural anesthesia; VAS, visual analog scale.

### Survival rate in the GA and GEA groups

According to survival curves, the survival rate of the GEA group was higher than that of the GA group (Figure 1). There was no significant difference observed regarding the 1-year survival rate between the two groups (*P*>0.05). From the second year onward, the survival rate of two groups began to decrease. A significant difference in relation to the 5-year survival rate as well as a 95% confidence interval (CI) was detected between the two groups (*P*<0.05, Table 9).

**Figure 1:** Survival rate curves of patients in the GA and GEA groups Notes: The upper curve, the survival curve of the combined general/epidural anesthesia group; the survival curve of the lower curve, the general anesthesia group; +, cencored; GA, general anesthesia; GEA, combined general/epidural anesthesia.

**Table 9:** Comparisons of survival rates between the GA and GEA groups

Time	Group	Survival rate (95% CI)	*P*
1 year	GA group	96.8 (56.23–60.44)	0.412
	GEA group	98.4 (57.75–60.34)	
2 years	GA group	91.9 (52.46–58.36)	0.635
	GEA group	93.5 (52.91–58.55)	
3 years	GA group	77.4 (43.91–51.69)	0.389
	GEA group	82.3 (45.84–53.36)	
4 years	GA group	72.6 (41.76–49.65)	0.182
	GEA group	80.6 (44.92–52.61)	
5 years	GA group	60.5 (37.42–45.23*)	0.006
	GEA group	79.0 (44.56–52.17*)	

Notes: *, compared with the GEA group, *P*<0.05; Abbreviations: CI, confidence interval; GA, general anesthesia; GEA, combined general/epidural anesthesia.

## Discussion

During the study, the effects of GA and GEA on cellular immune function and the prognosis of OC patients undergoing tumor resection were investigated. We demonstrated that anesthesia could damage cellular immune function due to its postoperative analgesic effects and reduce the survival rate.

Our study detected the concentrations of immunologic factors such as TNF-α and IL-2 in serum, hence providing evidence that OC patients in the GEA group exhibited higher serum concentrations of IL-2 and TNF-α than those in the GA group. The proliferation and invasion of tumor cells is associated with the release of certain cytokines such as TNF-α and IL-2, which could induce immunosuppression by favoring tumor cell proliferation [16]. Zou et al. [17] reported that anesthesia harms the immune function of red blood cells in OC patients undergoing laparoscopic therapy. Evidence has recently emerged demonstrating that GEA might help improve the body’s defense against tumor progression more than GA in malignant patients [18]. Furthermore, our study demonstrated that RTRR, RRICR, and RRCR were much higher in the GEA group than in the GA group. It was also established during our study that the rosette of tumor cells could stick to red blood cells and inhibit the metastasis of tumor cells [19]. A further finding of our study was in relation to the detection of reduced expression of T-cell subsets (CD3^+^, CD4^+^, CD4^+^/CD8^+^, and CD8^+^) and NK cells (CD16^+^ and CD56^+^) in the GEA group in comparison with the GA group. Dong et al. [20] found that anesthesia can impair macrophage, neutrophil, T cells, NK cells, and dendritic cell functioning. Moreover, Sofra et al. [16] reported that T cells play a role in tumor suppression. NK cells are associated with tumor development in different cancers by detecting and destroying the circulation of tumor cells and providing critical host protection against tumor progression and metastasis. This can be attenuated by anesthesia [20]. Our results demonstrated that GEA had a relatively minor effect on the expression of T-cell subsets and NK cells (indicated by CD3^+^, CD4^+^, CD4^+^/CD8^+^, CD8^+^, CD16^+^, and CD56^+^) than GA. Generally speaking, it is reasonable to hypothesize that GEA affects cellular immune functioning less so than that of GA.

In regards to the prognosis of OC patients, our study found the GEA exhibited more stable hemodynamics, less pain, and higher survival rates. First, the hemodynamics parameters such as SBP, DBP, and HR of patients in the GA group at T1, T2, and T3 were significantly lower than those of patients in the GEA group. According to Bettex et al*.* [21], GA can cause hemodynamic instability and local anesthesia may provide more hemodynamic stability. Therefore, we felt it reasonable to arrive as the conclusion that GEA benefits hemodynamic stability. Second, the VAS score of the GEA group 72 h after operation was lower than that of the GA group, suggesting that GEA may perform better in relieving postoperative pain than that of GA. Similarly, Pei et al. [22] demonstrated that epidural anesthesia can provide much better pain relief postoperation, reserve the ability of immune response caused by the stress response leading to an overall better prognosis. Moreover, Khajavi et al. [23] reported that their requirement for analgesics were significantly reduced due to less pain experienced after a lumbar laminectomy procedure. Third, the 5-year survival rate of OC patients who were dosed with GEA was higher than those who received GA. Wang et al*.* [24] indicated that epidural anesthesia plays a role in prolonging the survival time of cancer patients. In addition, Sun et al. [25] found that epidural anesthesia can improve the overall survival rate of patients with colorectal cancer. In summary, patients treated with GEA had more positive outcomes than those treated with GA.

## Conclusion

The present retrospective analysis included 248 women suffering from OC, who underwent laparoscopic tumor resection. The trial demonstrated significant differences between patients receiving GEA and GA in terms of cellular immune functioning and prognosis. GEA appears to be more beneficial in maintaining cellular immune function, achieving a better prognosis thus offering a novel insight into the selection of clinical anesthesia. However, due to the relatively small sample size of our study, undue influence may have an impact on the prognostic outcomes. The present study was largely based on retrospective data whereby patients had received GA or GEA anesthesia were randomly divided into two groups from the population, and as a result lacking in randomized prospective study value. Therefore, further investigation with larger sample sizes and a greater number of anesthetic methods are required in future studies.

## Abbreviations

DBP: diastolic blood pressure
FITC: fluorescein isothiocyanate
GA: general anesthesia
GEA: general/epidural anesthesia
HR: heart rate
IL: interleukin
LSD: least significant difference
NK: natural killer
OD: optical density
OC: ovarian cancer
RRCR: rate of red cell C3b receptor rosette
RRICR: rate of red cell immune complex rosette
RTRR: rate of tumor-red cell rosette
SBP: systolic blood pressure
TNF-α: tumor necrosis factor-α
VAS: visual analog scale
